# Hsp72-Based Effect and Mechanism of Microwave Radiation-Induced Cardiac Injury in Rats

**DOI:** 10.1155/2022/7145415

**Published:** 2022-08-18

**Authors:** Dayan Li, Xinping Xu, Yabing Gao, Juan Wang, Yue Yin, Binwei Yao, Li Zhao, Haoyu Wang, Hui Wang, Ji Dong, Jing Zhang, Ruiyun Peng

**Affiliations:** Beijing Institute of Radiation Medicine, Beijing, China

## Abstract

The purpose of this study was to determine the role of heat shock protein 72 (Hsp72) changes in cardiac injury caused by microwave radiation, aimed at providing novel insights into the mechanism of this damage. A digital thermometer was used to measure the rectal temperature of the rats' pre- and post-radiation. On the 1^st^, 7^th^, 14^th^, and 28^th^ days post-radiation, the changes in electrocardiogram (ECG) were analyzed by a multi-channel physiological recorder. The myocardial enzyme activities and ion concentrations were detected by an automatic biochemical analyzer. Additionally, the levels of myocardial injury markers were established by the enzyme-linked immunosorbent assay (ELISA), and those of hormones were measured by radioimmunoassay. The structure and ultrastructure of the myocardial tissue were observed using an optical microscope and transmission electron microscopy (TEM). The expression of Hsp72 was measured by Western blot and immunofluorescence analyses. Post-exposure, the rectal temperature in the R-group increased significantly, ECG was disordered, and the concentrations of ions were decreased. Furthermore, the activities of myocardial enzymes were changed, and the contents of myocardial injury markers and hormones were increased. We observed damage to the structure and ultrastructure and significantly increased expression of Hsp72. As a whole, the results indicated that S-wave microwave radiation at 30 mW/cm^2^ for 35 min resulted in damage to the cardiac functionality organigram, caused by a combination of the thermal and nonthermal effects.

## 1. Introduction

Microwave technology has been increasingly used in wireless communication and research fields in medicine, but excessive human exposure and the accompanying risk of energy leakage require more attention [1]. A large number of studies have shown that microwave radiation exerts adverse effects on human health. The biological effects of electromagnetic radiation are classified as thermal and non-thermal effects. It is generally believed that the non-thermal effect refers to that alteration in the physiological process without increasing the temperature of the organism. The temperature changes pre- and post-radiation within 1°C are generally regarded as a non-thermal effect. The thermal effect indicates that the temperature increases after the organism absorbs electromagnetic energy, which causes a series of pathological changes [2]. The heart, as the circulatory power organ with the most abundant electrical signals, is also the most sensitive target organ affected by microwave radiation [3].

Currently, the research on microwave radiation-induced cardiac injury has also focused on the non-thermal effect [4]. Preliminary studies performed by our group have revealed that 15 min of S-band microwave radiation causes only the non-thermal effect, with slight damage and fast recovery [5]. The damage caused by the non-thermal effect of microwave radiation is manifested mainly in structural cardiac damage, changes in myocardial enzyme levels, and ion disorders [1]; these indicators have been used conventionally [6]. However, with the widespread application of S-wave in communications, people are exposed to the electromagnetic environment for increasingly longer durations [7], and thus, the thermal effect of microwave radiation is causing rising concerns. Currently, no report has been published on the thermal effect induced by microwave radiation in the S-wave, especially studies on cardiac damage. Therefore, we developed a thermal effect model by extending the irradiation time in this study. In terms of index selection, we selected the changes in the levels of myocardial enzymes (CK-MB and HBDH) [8] and myocardial injury markers (H-FABP, cTnT, and NT-pro BNP) [9, 10]. The reason behind our selection is that they are not only more closely related to clinical manifestations but are also more sensitive to myocardial injury than traditional myocardial enzymes such as AST. In addition, we also evaluated the endocrine and electrophysiological functions of the heart, detected the levels of cardiac-specific secreted hormones (ANP and ET) [11, 12], and systematically analyzed the ECG results. Compared with previous studies, the establishment of the thermal effect model and the selection of indicators in this study are innovative to a certain extent.

Heat shock proteins are a group of non-secreted proteins that can be newly synthesized or their levels increased by heat cell stress [13, 14]. Heat shock protein 72 (Hsp72) is a protein whose synthesis is easily induced by heat stress; it is involved mainly in the processes of clearing and repairing damage sites [15, 16]. Studies have shown that the protein is rarely expressed in the myocardium in the absence of heat stress, which can otherwise lead to its significant upregulation. Hsp72 may be involved in the regulation of ion concentration changes and the decrease in electrical remodeling alterations, resulting in the prevention or delay of the occurrence and development of atrial fibrillation [17]. The role of Hsp72 in heat stress has been elucidated; it regulates cardiac electrophysiological functions [18]. Therefore, in this study, we innovatively used this protein to create the thermal effect caused by microwave radiation, which would provide novel insights into the damage mechanism.

Accordingly, we applied S-band microwave exposure in a single 35 min irradiation treatment of rats to determine the damage effect. ECG and changes in the biochemical function and structure were employed to explore whether the changes induced were due to the combination of thermal and non-thermal effects.

## 2. Materials and Methods

### 2.1. Experimental Animals

The experiment was approved by the Animal Ethics Committee of the Beijing Institute of Radiation Medicine. Fifty male Wistar rats (weighing 280 ± 20 g) were purchased from Beijing Charles River Center for Experimental Animals. The rats were fed in a laboratory facility that met SPF standards (22 ± 1°C, a standard rodent diet ad libitum; 12 h light/12 h dark cycle; three rats were kept per cage). Approval for the experiments was obtained from the Academy of Military Medical Sciences' ethical committee (approval number: IACUC-DWZX-2021-650). All surgeries were performed under 1% sodium pentobarbital anesthesia.

### 2.2. Groups and Microwave Exposure

Fifty rats were weighed and randomly split into two groups of equal size using the stratified random method to eliminate the impact of body weight. The following groups were assigned: radiation (2.856 GHz microwave exposure) group (R group) and control group (C group). Each group was composed of 25 rats. Five of these 25 rats in each group were used for electrophysiological experiments, and 20 were used for blood and heart collection on the 1^st^, 7^th^, 14^th^, and 28^th^ days post-radiation, with five rats at each time point.

A microwave radiation source developed by the Academy of Military Medical Sciences was applied to conduct uniform radiation throughout the body. The rats were placed in a self-made radiation box. The radiation box was made of acrylic without metal substances, with ventilation holes evenly distributed on the surface. The rats were fixed in the radiation box with their heads facing the center of the disk. The radiation disk was placed in an irradiation chamber filled with absorbing material, and the rats were exposed to the exposure table directly below the radiation source. The exposure table was rotated to eliminate positional effects. The rats in the R group were irradiated by 30 mW/cm^2^ S-band microwave exposure for 35 min. The rats in the C group were also placed in the radiation box and on the radiation table but were not irradiated (Figure 1).

Five rats were randomly chosen from each group, and the intellectual digitizing thermometer was used to measure the core temperature before and immediately after the radiation treatment (Zhongwang, Beijing).

### 2.3. ECG Examination

A multi-channel physiological recorder (BIOPAC, USA) was utilized to track the ECG of the rats at the four experimental post-radiation time points. Each group contained five rats. After weighing, the rats were intraperitoneally administered with 1% pentobarbital sodium (1 mL/100 g). The rats' limbs were then sheared, impaled in a supine posture, and cleaned. Additionally, red wire electrodes were inserted into the subcutaneous tissue of the right upper limb, black wire electrodes into the right lower limb, and green wire electrodes into the left lower limb, all of which were coupled to an ECG bio-amplifier at a sensitivity of 2000 Hz. Next, the rats were kept in complete silence to record for 3 min. Finally, we analyzed and computed the changes in the R, P, and T-waves and the heart rate.

### 2.4. Serum Biochemical Analysis

Five rats from each group were subjected to the procedure described in Materials and Methods, Sub-section 2.3 at the four experimental time points. After the rats were put in slumber, 3 mL of blood was taken from the inferior vena cava (IVC) to produce serum. The activities of AST, CK, LDH, CK–MB, and HBDH and the concentrations of K^+^, Na^+^, Cl^−^, and Ca^2+^ were detected by an automated biochemical analyzer (Coulter JTIR, USA).

### 2.5. Content of Myocardial Injury Markers

Five rats from each group were taken at the four experimental time points post-radiation. Following anesthesia of the rats (the procedure was identical to that reported in Materials and Methods, Sub-section 2.3), 3 mL of blood was taken from the IVC to produce serum. The contents of cTnT, H-FABP, and NT-pro BNP in the serum were estimated using an ELISA kit (FuruiRunze, China). The steps were as follows: (1) the diluted gradient standard was added to the ELISA-coated plate. (2) The serum was added to the ELISA-coated plate; then, the enzyme labeling reagent was added except for the blank wells, incubated for 30 min (37°C), and washed with PBS with 0.05% Tween (TBST) five times. (3) Color developer buffer was added to each well, mixed, and avoided light at 37°C for 15 min. (4) We then added a stop buffer, measured the optical density (OD) value of each well at 450 nm with a microplate reader within 15 min, and calculated the contents of cTnT, H-FABP, and NT-pro BNP in the rats' serum by the OD value.

### 2.6. Detection of the Hormone Content

Five rats from each group were taken at the four experimental time points post-radiation. Following anesthesia of the rats (the exact procedure is identical to that described in Materials and Methods, Sub-section 2.3), 3 mL of blood was taken to produce serum from the IVC. Following the instructions of the manufacturer of the radioimmunoassay kit (FuruiRunze, China), the following procedure was employed: (1) we quantitatively added the antigen (standard substance and serum to be tested), labeled the antigen and antibody to the cuvette in sequence, mixed well, and reacted at a suitable temperature for an appropriate time. (2) Next, we added PR reagent for separation, mixed, and put the samples to room temperature. (3) Further, we performed centrifugation at 4°C and 3500 r for 20 min, discarded the supernatant, measured the number of precipitated cpm, and calculated the contents of ANP and ET.

### 2.7. Structure of Rats' Myocardial Tissue

We anesthetized five rats from each group, selected them randomly at the four experimental time points post-radiation, and removed their hearts. The hearts were immersed in pre-cooled normal saline and rinsed until no residual blood was present. Next, we divided each heart into two parts, and the right half was cryopreserved, while the left half was fixed in a 10% formalin fixative solution for at least a week. The paraffin-embedded cardiac tissues were cut into 5-*μ*m slices after dehydration, tissue transparency, and immersion in wax. After being dewaxed and dried (60°C) for 48 h, the tissues were stained with the haematoxylin and eosin stain. A microscope (Leica, Germany) was used to view and snap photos of the dyed slices.

### 2.8. Ultrastructure of Rats' Myocardial Tissue

Three rats from each group were taken at the four post-radiation experimental time points, and their hearts were extracted while the animals were sedated. Approximately 1 mm^3^ of fresh tissue piece was taken from the cardiac apex, fixed in 2.5% glutaraldehyde for 2 h, and deposited in 1% osmic acid fixative for 1 h. Then, it was dehydrated with gradient ethanol, transferred with acetone, and implanted into Epon 812 resin. To determine the location of the most serious damage, the tissues were sliced into semithin sections. After cutting into 70 nm ultrathin slices, the semithin slices were dyed with lead-uranium, observed, and photographed by TEM.

### 2.9. Expression of Hsp72 in Rats' Myocardial Tissue

The frozen cardiac tissue collected at the four experimental post-radiation time points was subjected to Western blotting. The treatment procedures were as follows: 20 mg of each frozen myocardial tissue was removed, followed by the addition of 200 *μ*L of tissue lysis buffer at a ratio of 1 mg/10 mL (protease inhibitor : lysate = 1 : 100). The appropriate number of magnetic beads was next added, and the mixture was automatically homogenized ten times at 60 Hz, 45 s each time (at 15 s intervals). Then, it was soaked for 10 min in ice and centrifuged at 12,000 r/min for 15 min at 4°C). The supernatant was collected, and the bicinchoninic acid protein measurement kit was used (Thermo, USA). Protein and loading buffer were mixed at a ratio of 4 : 1 and heated at 95°C for 10 min, and then, the sample was cooled down and subjected to SDS-PAGE.

After electrophoresis, membrane transfer, and blocking, the mouse anti-Hsp72 (TBST diluted to 1 : 1000; Enzo Life Sciences, USA) and the rabbit anti-GAPDH (TBST diluted to 1 : 10,000; Abcam, USA) were added, shaken slowly for an entire night in a shaker (4°C), and washed with TBST three times. HRP-labeled goat anti-mouse IgG (TBST diluted to 1 : 10,000; Beyotime, China) was then added, shaken for an hour at room temperature, and washed with TBST three times. The unclear bands were rejected if the bands of Hsp72 or the bands of GAPDH were incomplete, whereas the clear bands were semiquantified by their OD values. Statistical analysis was carried out after the Western blotting experiments were repeated at least three times.

### 2.10. Expression and Distribution of Hsp72 in Rats' Myocardial Tissue

On the 1^st^, 7^th^, 14^th^, and 28^th^ days post-radiation, half of the myocardia were subjected to immunofluorescence analysis. The steps before drying the slices at 60°C for two days are the same as those described in Materials and Methods, Sub-section 2.7. The operation steps were as follows: dewaxing by xylene, antigen retrieval, threefold washing with PBS, and blockage with 10% goat serum for 1 h. Then, mouse anti-Hsp72 (10% goat serum diluted at 1 : 75; Enzo Life Sciences, USA) was added, and the specimens were incubated overnight in a humidified box at 4°C, rewarmed at room temperature for an hour, and washed with PBS three times. Further, fluorescent-labeled goat anti-mouse IgG (10% goat serum diluted at 1 : 100; Beyotime, China) was added, and the samples were incubated at room temperature for an hour in the dark, washed with PBS three times, and slip-covered with antifluorescence quenching solution containing DAPI. Finally, we performed observations and took photographs with a laser confocal microscope (Nikon, Japan), processed semiquantitatively by ImageJ, and performed the statistical analysis.

### 2.11. Experimental Program and Statistical Analysis

In this study, four time points were set at 1^st^, 7^th^, 14^th^, and 28^th^ post-exposure. Post-radiation, core temperature measurement, HE staining, transmission electron microscopy, serological examinations (myocardial enzymes, myocardial injury markers, ions, and hormones), ECG examination, and Western blotting were performed to comprehensively evaluate the cardiac damage. The corresponding relationship between the experimental procedure steps and time is illustrated in Figure 2.

The data of this paper are expressed as mean ± SD (*X* ± *S*) and compared with those of the C group. Statistical analysis was carried out using SPSS 19.0 version and an independent sample *t*-test. The acceptable significance level of all trials was set at *P* < 0.05. On the basis of the *P*-value, the significance was classified as: ^∗^*P* < 0.05 and ^∗∗^*P* < 0.01.

## 3. Results

### 3.1. Microwave Radiation Increased Core Temperature

Compared with the C group, the core temperature post-radiation in the R group was observably higher than that before radiation (*P* < 0.01), and the average value rose above 2.3°C (Figure 3). The biological effect of this experiment may be due to the combination of the thermal and non-thermal effects, which needs to be verified in combination with other detection indicators.

### 3.2. Microwave Radiation Led to ECG Result Disorder

Compared with the C group, the heart rate of the R group was significantly higher on the 1^st^, 7^th^, and 14^th^ days post-radiation (*P* < 0.05 or 0.01), but with no significant difference on the 28^th^ day post-exposure (*P* > 0.05) (Figure 4); the amplitude of the P-wave in the R group was significantly increased on the 1^st^ and 7^th^ days post-radiation (*P* < 0.05 or 0.01), but no remarkable difference was observed on the 14^th^ and 28^th^ days post-radiation (*P* > 0.05) (Figure 5). The P-wave duration in the R group was significantly shorter than that in the C group on the 1^st^ and 7^th^ days post-radiation (*P* < 0.05), with no prominent difference on the 14^th^ and 28^th^ days post-radiation (*P* > 0.05) (Figure 6). Compared with the C group, the amplitude of the R-wave in the R group was significantly increased on the 7^th^ day post-radiation (*P* < 0.05), but there was no noteworthy difference at other time points (*P* > 0.05) (Figure 7). The T-wave amplitude in the R group was significantly lower than that in the C group on the 1^st^ and 7^th^ days post-radiation (*P* < 0.05 or 0.01), but no remarkable difference was detected on the 14^th^ and 28^th^ days post-radiation (*P* > 0.05) (Figure 8).

The aforementioned results showed that the electrophysiological function of the rat heart was significantly damaged on the 1^st^ and 7^th^ days post-exposure, and the heart rate did not recover until the 14^th^ day post-radiation.

### 3.3. Microwave Radiation Changed Serum Biochemical Function

#### 3.3.1. Changes in Myocardial Enzyme Activity

The activities of AST, LDH, and CK were observably increased in the R group as compared with those in the C group on the 1^st^ day post-radiation (*P* < 0.05 or 0.01); there was no noteworthy difference on the 7^th^, 14^th^, and 28^th^ days post-exposure (*P* > 0.05) (Figures 9(a)–9(c)); the activities of CK-MB and HBDH on the 7^th^ day post-radiation were significantly decreased (*P* < 0.01), and there was no discernible difference between the two groups at other time points (*P* > 0.05) (Figures 9(d) and 9(e)). We speculated that the changes in myocardial enzyme activity might have been caused by the damage in the myocardial cell membrane, which had induced the leakage of myocardial enzymes in the myocardial cells.

#### 3.3.2. Ion Concentration Decreased

The concentrations of K^+^ and Na^+^ in the R group were significantly lower than those in the C group, but on the 1^st^ day post-exposure (*P* < 0.01), there was no remarkable difference from those detected at the other time points (*P* > 0.05) (Figures 10(a) and 10(b)); the concentrations of Ca^2+^ in the R group were observably decreased on the 1^st^ day post-radiation (*P* < 0.01) and increased on the 7^th^ and 14^th^ days post-radiation (*P* < 0.05 or 0.01); there was no prominent difference on the 28^th^ day post-radiation (*P* > 0.05) (Figure 10(c)). The concentrations of Cl^−^ in the R group were significantly lower on the 1^st^, 7^th^, and 14^th^ days post-radiation (*P* < 0.05), but there was no noteworthy difference on the 28^th^ day post-radiation (*P* > 0.05) (Figure 10(d)). The overall changes in the serum ion concentration in the serum showed a downward trend, presumably because of the rats' dehydration due to the thermal effect post-exposure.

### 3.4. Microwave Radiation Increased the Level of Myocardial Injury Markers

The cTnT concentrations in the R group at the four experimental time points post-radiation were significantly higher (*P* < 0.01) than those in the C group (Figure 11(a)). The concentrations of NT-pro BNP on the 1^st^, 7^th^, and 14^th^ days post-radiation were significantly higher (*P* < 0.05 or 0.01), but there was no significant change on the 28^th^ day post-radiation (*P* > 0.05) (Figure 11(b)). The concentration of H-FABP was significantly higher only on the 7^th^ day post-exposure (*P* < 0.05), whereas no noteworthy differences were observed at the other time points (*P* > 0.05) (Figure 11(c)). The levels of myocardial injury markers in the serum were all increased, which further confirmed that the myocardial function was seriously damaged. Additionally, cTnT and NT-pro BNP recovered slowly, indicating that they can reflect myocardial injury more sensitively than myocardial enzymes.

### 3.5. Microwave Radiation Increased the Level of Hormones

Compared with the C group, the contents of ANP in the R group were significantly higher at the four experimental time points post-radiation (*P* < 0.05 or 0.01) (Figure 12(a)). The contents of ET were significantly higher only on the 14^th^ and 28^th^ days post-radiation (*P* < 0.05 or 0.01) but had no significant change on the 1^st^ and 7^th^ days post-radiation (*P* > 0.05) (Figure 12(b)). The contents of ANP and ET reflect the endocrine function of the heart [19] and can affect many functions of the organism [20]. In this experiment, the contents of ANP and ET were significantly increased, which may be the reason for the cardiac electrical disturbance and ion concentration changes established.

### 3.6. Microwave Radiation Induced Myocardial Structure Abnormalities

Considering the results of our prior experiment, the rats' cardiac function damage did not recover within 14 d post-radiation. Therefore, in this experiment, we selected the 1^st^, 7^th^, 14^th^, and 28^th^ days as the time points of tissue structure observation to elucidate the time-varying laws of cardiac tissue structural damage post-radiation.

Within the 28^th^ day post-radiation, the endothelial cell nuclei were fusiform; the myocardial cells were oval, and the myocardial fibers were neatly aligned in the C group (Figure 13(a)). On the 1^st^ day post-exposure, myocardial fiber arrangement disorder and pyknotic hyperstaining appeared in the R group (Figure 13(b)). On the 7^th^ day post-exposure, cells were deformed and shed, and nucleus pyknosis hyperstained into sheets (Figure 13(c)). On the 14^th^ day post-radiation, the rats' myocardial fiber arrangement was wavy, and the myocardial cells were edematous, but pyknosis and hyperchromasia were relieved (Figure 13(d)). On the 28^th^ day post-exposure, it was basically recovered (Figure 13(e)). The above results showed that the most significant time points for tissue structural damage in this model are the 1^st^ and 7^th^ days post-exposure, and there was a recovery trend on the 14^th^ and 28^th^ days post-exposure. The time-varying laws of myocardial tissue structure and cardiac function damage were basically consistent.

### 3.7. Microwave Radiation Led to Abnormal Myocardial Ultrastructure

Through the comprehensive analysis of the aforementioned results, in this study, we selected the 1^st^, 7^th^, 14^th^, and 28^th^ days as the time points of myocardial tissue ultrastructure observation to clarify the different time-varying laws of the ultrastructure indifferent injury sites post-exposure.  Figure 14-a, b, and c depict the changes in the myocardial fibers, mitochondria, and nuclei, respectively.

Within 28 days post-radiation, the myocardial fibers in the C group were arranged neatly, and the Z line was straight and clear, as observed under an electron microscope (Figure 14(a)-A). In the R group, on the 1^st^ day post-radiation, the myocardial fibers were loosely arranged, the myofilaments were blurred and dissolved, and the Z line was distorted (Figure 14(a)-B). On the 7^th^ day post-exposure, the myocardial fiber damage was the most serious, considerable segmental dissolution; the Z line was broken and blurred (Figure 14(a)-C). On the 14^th^ day post-exposure, myocardial fiber damage had begun to recover but was still dissolved to some degree, while the Z line was intact but slightly curved (Figure 14(a)-D). Then, on the 28^th^ day post-exposure, the myocardial fiber injury was basically recovered (Figure 14(a)-E).

Within 28 days post-exposure, the mitochondria in the C group were more numerous and structurally intact in our observations under an electron microscope (Figure 14(b)-A). In the R group, on the 1^st^ day post-exposure, the mitochondria were swollen and cavitated seriously; their number was reduced, and their shape and size were different (Figure 14(b)-B). On the 7^th^ day post-exposure, the mitochondria were damaged and with more cavitation (Figure 14(b)-C). Later, on the 14^th^ day post-exposure, the mitochondria still had a small amount of cavitation, and the cristae were unclear, but a slight recovery was observed (Figure 14(b)-D). On the 28^th^ day post-exposure, the mitochondrial damage was basically recovered (Figure 14(b)-E).

Our observation under an electron microscope showed that the karyotype of the C group was regular within 28 days post-exposure (Figure 14(c)-A). In the R group, on the 1^st^ day post-exposure, the perinuclear space was slightly widened, and the chromatin margins were gathered (Figure 14(c)-B). On the 7^th^ day post-exposure, the perinuclear gap widened further, and the chromatin margins were additionally gathered, showing that the most serious nuclear damage was established on the 7^th^ day post-exposure (Figure 14(c)-C). On the 14^th^ day post-exposure, the perinuclear space and the nuclear damage had begun to recover (Figure 14(c)-D). Then, on the 28^th^ day post-radiation, the karyotype was regular, and the nuclear damage was completely recovered (Figure 14(c)-E).

In this study, electron microscopy was used to observe the damage to the myocardial fibers, mitochondria, and nuclei in the cardiomyocytes. We found that the time-varying laws of different ultrastructural sites were basically consistent and in agreement with the temporal changes in cardiac function and myocardial tissue structural damage. The most significant injury was established on the 1^st^ and 7^th^ days; the recovery trend appeared on the 14^th^ day post-radiation.

### 3.8. Microwave Radiation Increased the Hsp72 Expression

On the 1^st^ and 7^th^ days post-exposure, the rats' cardiac expression of Hsp72 in the R group was significantly higher than that in the C group (*P* < 0.05 or 0.01), especially on the 1^st^ day post-radiation. On the 14^th^ and 28^th^ days post-exposure, there was no remarkable change in the Hsp72 expression in the rat myocardial tissue (*P* > 0.05) (Figure 15). The increase in the Hsp72 expression was consistent with the results of the core temperature, which suggested that the model was caused by the combination of the thermal and non-thermal effects.

The Western blotting results showed that on the 1^st^ and 7^th^ days post-radiation, the Hsp72 of the R group was significantly increased. Therefore, in this experiment of immunofluorescence, we selected the 1^st^ and 7^th^ days as time points with the most obvious changes.

Under a laser confocal microscope, we found that Hsp72 in the myocardial tissue of the C group had almost no expression, whereas Hsp72 in the R group was abundant in the nucleus and cytoplasm. The statistical analysis conducted revealed that the expression of Hsp72 in the R group was significantly higher than that in the C group on the 1^st^ and 7^th^ days post-radiation (*P* < 0.01) (Figure 16). The increase in the Hsp72 expression in rats' myocardia was consistent with the results of core temperature and Western blotting. Therefore, we again confirmed that the changes in the model were caused by the combination of the thermal and non-thermal effects, indicating that the bioeffect of microwave radiation was time-dependent.

## 4. Discussion

The heart is the power organ in the circulatory system, which delivers nutrients and eliminates metabolic waste through its contraction and relaxation. It is also one of the most sensitive organs to electromagnetic radiation. Microwave radiation can affect both the function and the structure of the heart. Previous research conducted by our group has examined mainly the non-thermal effect of microwave radiation exerted for less than 15 min. In this study, 25 rats were irradiated by an S-band microwave for 35 min. Nine rats in the R group were paralyzed and unable to stand upright and walk normally, while two rats in this group died. By comparing the previous research of our group, we found that the rats' state was completely different from that established in the experiment in which the radiation time was less than 15 min, although the same radiation dose was applied. Therefore, we speculate that the changes in the aforementioned rat vital signs may be closely related to the irradiation time used in this experiment.

Electrocardiography is an objective approach to evaluating the electrophysiological function of the heart. Numerous studies have shown that microwave radiation can lead to changes in ECG. Yan et al. [21] used microwaves with average power densities of 100 mW/cm^2^ and 200 mW/cm^2^ to irradiate New Zealand rabbits for 20 min. After the rabbits were irradiated at 100 mW/cm^2^ for 15 min, the R-wave and QR-wave were abnormal. Based on this previous evidence, in this study, we intended to judge the effect of microwave radiation on cardiac electrophysiological function by the assessment of ECG results of the experimental rats. Our results showed that the cardiac conduction function was seriously damaged on the 1^st^ and 7^th^ days post-exposure, and the change in the heart rate was not recovered until the 14^th^ day post-exposure, manifested as an increase in heart rate, increased P-wave amplitude, decreased P-wave duration, increased R-wave amplitude, and decreased T-wave amplitude. These postirradiation outcomes might have been caused by the increase in the body temperature, the abnormal dynamics of important ions in the blood, and the dehydration of the rats.

After myocardium damage or necrosis, myocardial enzymes are released into the blood. Thus, to evaluate the injury, it is necessary to detect the levels of myocardial enzymes and ions in the serum. A number of studies have shown that microwave radiation can lead to disturbances of ion concentrations and myocardial enzyme activities in the serum [6, 21]. In this study, serum biochemical analysis revealed damage on the 1^st^, 7^th^, 14^th^, and 28^th^ days post-exposure. The concentrations of K^+^, Na^+^, and Cl^−^ were significantly decreased, while the concentrations of Ca^2+^ decreased significantly on the 1^st^ day post-exposure and then increased significantly on the 7^th^ and 14^th^ days post-exposure. We speculated that the changes in the serum ions post-radiation might be related to dehydration, affecting the excitability of cardiomyocytes, thereby causing changes in the rhythm of cardiomyocytes. This notion may explain the longer duration of ECG disturbances and the slower recovery in this study than those in previous. The results of myocardial enzymes showed that the rat myocardium was severely damaged, suggesting that the structure of the myocardial cell membrane may be damaged, resulting in the release of myocardial enzymes into the blood.

Furthermore, in the exploration of cardiac injury biological indicators, in addition to serum ions and enzymes, indicators such as cTnT, H-FABP, and NT-pro BNP are widely used in cardiac disease screening [22]. Our review of the relevant research literature showed that cTnT, H-FABP, and NT-pro BNP changed earlier and were more sensitive than myocardial enzymes after cardiac function damage, which are precise indicators for cardiac function evaluation. Jo et al. [23] established that H-FABP was significantly increased in the early stage of myocardial injury and concluded that it could be combined with myocardial enzymes, ANP and ET, for myocardial injury diagnosis. Suthahar et al. [24] revealed that cTnT and NT-pro BNP were significantly correlated with myocardial injury. In this investigation, we found that microwave radiation significantly increased the contents of cTnT, H-FABP, and NT-pro BNP. Moreover, we confirmed that myocardial injury occurred on the 1^st^ day post-exposure, and myocardial injury was not completely recovered on the 28^th^ day post-exposure. The changes in the levels of the serum myocardial injury markers in the present study suggest that they can be more sensitive to indicate myocardial injury than other indicators. In this model, the sensitivity to a myocardial injury can be ranked in the following descending order: cTnT > NT − pro BNP > H − FABP.

A large number of recent studies have shown that ANP and ET are closely related to cardiac function. Unlike other hormones, they are synthesized and secreted by the heart, which can reflect changes in cardiac endocrine function [25]. ANP and ET can maintain normal cardiovascular contraction and material exchange, regulating serum ion concentrations and cardiac electrical activity [26, 27]. In related research on microwave radiation effects, microwave exposure at 30 mW/cm^2^ changed the contents of ET and ANP in rats' serum [27]. In this study, we found that ANP and ET levels in the serum increased post-radiation and did not recover on the 28^th^ day post-exposure, which was consistent with the results of myocardial injury markers. Severe damage occurred in the model animals used in this investigation, and their recovery speed was low. Based on the physiological functions of ANP and ET, we speculated that the changes in ANP and ET may be an important material basis for the alterations in the ion concentrations and the ECG disturbance in this model.

The aforementioned results show that the heart function of the rats in this model was damaged, while it is known that functional changes and structural damage are frequently interrelated. Koniari et al. [27] and Yin et al. and Zhang et al. [28, 29] found that 7–30 days after microwave irradiation of rats at 2.5, 5, 10, and 50 mW/cm^2^, the myocardial fibers' arrangement was disordered, the structure of the intercalated discs was blurred, the mitochondria were swollen and cavitated; the increase in the radiation dose aggravated the existing lesions. In this study, the rats' myocardial structure and ultrastructure were observed under an optical microscope and transmission electron microscope, respectively. Our observations confirmed that the damage was significant on the 1^st^ and 7^th^ days post-exposure, slightly recovered on the 14^th^ day, and completely recovered on the 28^th^ day. The following manifestations were observed under the optical microscope: the myocardial fibers were disordered and wavy, and the nuclei were condensed and stained; under the electron microscope, we found that the myocardial fibrosis was dissolved, the Z line was broken and blurred, the mitochondria were swollen and cavitated, and the circumferential gap had been widened. The time-varying laws of myocardial structural damage were generally consistent with the results of most of the other indicators assessed in this study.

Therefore, our findings indicate that the exposure of rats to 30 mW/cm^2^ of S-band microwave radiation for 35 min can lead to cardiac functional and structural impairments. Part of the cardiac function was still not recovered on the 28^th^ day post-exposure. The above adverse changes were more serious, and the recovery was slower as compared to the damage caused by radiation exposure for 15 min, indicating that this effect was time-dependent.

The changes in the core temperature are within 2.3°C, which has exceeded the temperature change range of non-thermal effect in electromagnetic radiation (<1°C). We preliminarily speculated that this radiation could have a thermal effect, but the material basis and the related injury mechanism need to be verified. Hsp72 is the most sensitive heat shock protein to heat stress, and the changes in Hsp72 expression are manifested by certain indications for the occurrence of the thermal effect exerted by microwave radiation [30]. In this regard, Christian et al. [31] found that when the body was exposed to high temperatures, thermal excitation induced Hsp72 synthesis. Additionally, Wei [17] found that in animal experiments with rabbits, atrial Hsp72 expression was upregulated by heat stress, shortening the effective refractory period and frequency adaptation of the myocardium. Other researchers also found that Hsp72 regulated cardiac electrical disturbances by controlling the changes in ion concentration and reducing electrical remodeling alterations [17]. Our Western blotting and immunofluorescence experiments showed that the Hsp72 expression was significantly increased on the 1^st^ day post-exposure, which was consistent with the results of the core temperature. These data suggested that the cardiac injury in rats caused by radiation may be closely associated with the duration of their microwave radiation exposure.

To sum up, in this experiment, we simulated the working environment of occupational groups exposed to long-term electromagnetic irradiation. The animal model of long-term exposure of 35 min was used to systematically observe the vital signs and the cardiac structural and functional changes in the experimental rats. Our results showed that the cardiac function was abnormal, and myocardial structural damage occurred. Since the core temperature of the rats immediately increased post-radiation significantly, we further analyzed the expression of myocardial Hsp72. We preliminarily confirmed that the rat heart injury and heat stress model was successfully established after S-band microwave radiation through the significant increase in myocardial Hsp72 expression. Based on the findings obtained by the application of this model, this experiment provides novel insights into the damage mechanism of the thermal effect of microwave radiation, suggesting a new intervention target for research on protective measures.

## Figures and Tables

**Figure 1:** Diagram of the radiation devices employed in the experiments.

**Figure 2:** Schematic diagram of time arrangement.

**Figure 3:** Changes in rats' post-radiation anal temperature.

**Figure 4:** Changes in rats' ECG post-radiation: (a) records of ECG on the 1^st^, 7^th^, 14^th^, and 28^th^ days post-exposure; (b) heart rate analysis.

**Figure 5:** Changes in rats' ECG post-radiation: (a) changes in P-wave amplitude (the dashed frames refer to the P-wave); (b) P-wave amplitude analysis.

**Figure 6:** Changes in rats' ECG post-radiation: (a) changes in P-wave duration (the arrowheads refer to the P-wave); (b) P-wave duration analysis.

**Figure 7:** Changes in rats' ECG post-radiation: (a) changes in T-wave (the dashed frames refer to the T-wave); (b) T-wave amplitude analysis.

**Figure 8:** Changes in rats' ECG post-radiation: (a) changes in R-wave (the dashed frames refer to the R-wave); (b) R-wave amplitude analysis.

**Figure 9:** Changes in rats' myocardial enzyme activity in the serum post-radiation: (a) AST activity; (b) LDH activity; (c) CK activity; (d) CK-MB activity; (e) HBDH activity.

**Figure 10:** Changes in serum ion contents of rats in the serum post-radiation: (a) K^+^ concentrations; (b) Na^+^ concentrations; (c) Ca^2+^ concentrations; (d) Cl^−^ concentrations.

**Figure 11:** Changes in myocardial damage marker contents of rats in the serum post-radiation: (a) cTnT contents; (b) NT-pro BNP contents; (c) H-FABP contents.

**Figure 12:** Changes in ANP and ET contents of rats in the serum post-radiation: (a) ANP contents; (b) ET contents.

**Figure 13:** Changes in rats' myocardial structure post-radiation: (a) C group; (b) R group on the 1^st^ day; (c) R group on the 7^th^ day; (d) R group on the 14^th^ day; (e) R group on the 28^th^ day. (a–e) ×400, scale bar = 50 *μ*m (black frame indicates wavy fibers and injured parts).

**Figure 14:** Changes in rats' myocardial ultrastructure of post-radiation (scale bar = 500 nm): (a) myocardial fiber; A: C group on the 1^st^, 7^th^, 14^th^, and 28^th^ days (×10,000); B: R group on the 1^st^ day (×8000); C: R group on the 7^th^ day (×10,000); D: R group on the 14^th^ day (×10,000); E: R group on the 28^th^ day (×15,000). (b) Mitochondrion; A: C group on the 1^st^, 7^th^, 14^th^ and 28^th^ days (×25,000); B: R group on the 1^st^ day (×20,000); C: R group on the 7^th^ day (×25,000); D: R group on the 14^th^ day (×25,000); E: R group on the 28^th^ day (×25000). (c) Nucleus; A: C group on the 1^st^, 7^th^, 14^th^, and 28^th^ days (×10,000); B: R group on the 1^st^ day (×10,000); C: R group on the 7^th^ day (×15,000); D: R group on the 14^th^ day (×10,000); E: R group on the 28^th^ day (×12,000).

**Figure 15:** Changes in Hsp72 expression in rats' myocardial tissue post-radiation: (a) changes in Hsp72 expression; (b) analysis of the Hsp72 expression.

**Figure 16:** Changes in Hsp72 expression and distribution in rats' myocardial tissue post-radiation: (a) changes in Hsp72 expression and distribution (the line frames show the magnified figure; the arrows show positive signals); (b) analysis of the Hsp72 expression.

## Data Availability

The original contributions to the study are included in the Supplementary Material. Further inquiries can be directed to the corresponding author.
